The article "Clinical Efficacy of Assisted Reproductive Technology Combined with Progesterone Capsules in the Treatment of Infertility Caused by Diminished Ovarian Reserve and Its Influence on Serum FSH, E2, and LH Levels of Patients" was retracted in 2023. Reason: concerns about the peer review.

# Clinical Efficacy of Assisted Reproductive Technology Combined with Progesterone Capsules in the Treatment of Infertility Caused by Diminished Ovarian Reserve and Its Influence on Serum FSH, E_2_, and LH Levels of Patients

**DOI:** 10.1155/2022/5319172

**Published:** 2022-03-24

**Authors:** Lingqin Chen, Mindong Lai, Xiaojin Huang, Fang Zeng, Wei Xia, Qingping Yang, Sisun Liu

**Affiliations:** ^1^Department of Reproductive, The First Affiliated Hospital of Nanchang University, Nanchang 330006, Jiangxi Province, China; ^2^Medical Section, Jiangxi Cancer Hospital, Nanchang 330029, Jiangxi Province, China; ^3^Department of Obstetrics and Gynecology, The First Affiliated Hospital of Nanchang University, Nanchang 330006, Jiangxi Province, China

## Abstract

**Objective:**

To explore the clinical efficacy of assisted reproductive technology (ART) combined with progesterone capsules in the treatment of infertility caused by the diminished ovarian reserve (DOR) and its influence on serum FSH, E2, and LH levels of patients.

**Methods:**

In the manner of retrospective study, the data of 120 patients with infertility caused by DOR admitted to our hospital (February 2019–February 2020) were retrospectively analyzed, and the patients were equally divided into the experimental group and the control group according to the order of admission. All patients underwent in vitro fertilization and embryo transfer (IVF-ET), and the experimental group was received progesterone capsules at the same time. Ovarian-related indexes, follicular development, serum hormone levels, and pregnancy outcomes were compared between both groups.

**Results:**

After treatment, compared with the control group, ovarian-related indexes and follicular development in the experimental group were conspicuously better (*P* < 0.001). In the experimental group, the FSH level was (5.99 ± 1.20) U/L, the E_2_ level was (540.12 ± 3.54) ng/L, and the LH level was (3.10 ± 0.35) U/L after treatment, which was significantly better than those of the control group (*P* < 0.001). After treatment, compared with the control group, the clinical pregnancy rate in the experimental group was conspicuously higher (*P* < 0.05), and the abortion rate in the experimental group was conspicuously lower (*P* < 0.05). No obvious difference was observed in multiple births rate between the two groups (*P* > 0.05).

**Conclusion:**

ART combined with progesterone capsules can improve serum hormone levels, ovarian function, follicular development, and clinical pregnancy rate for patients with infertility caused by DOR, which should be applied in practice.

## 1. Introduction

Ovarian reserve function is to produce ovum of high quality and large quantity, which can fully reflect women's fertility. Nowadays, delayed childbearing in women has become the trend of population development, and more and more patients have diminished ovarian reserve (DOR) [1], presenting with sex hormone disorders, which disturbs the developmental ability of oocytes. As a result, their ability to produce high-quality oocytes is reduced, which leads to a decline in the number of follicles in their ovaries and a consequent increase in the incidence of infertility [2]. At present, drug treatment is the main method of infertility caused by DOR [3], like progesterone, and the patients desiring pregnancy are given estrogen and progesterone cyclical treatment. The drug treatment has delivered results to some extent, but patients are prone to suffer from breast pain, obesity, and other adverse reactions [4], and some patients also have symptoms such as oligomenorrhea after treatment with a high recurrence rate of the disease [5, 6]. With the continuous progress of assisted reproductive technology (ART), IVF-ET has been applied in infertility caused by endometriosis, polycystic ovary syndrome (PCOS), and other diseases, with the pregnancy rate reaching more than 40% [7–9]. However, according to many studies, the patients with DOR have a poor response to IVF-ET drugs and lack sensitivity, with a low clinical oocyte retrieval rate and a small number of high-quality embryos, so it is very important to apply safe and effective treatment to improve the quality of embryo and implantation rate. In the past ten years, natural progesterone has been widely used in the treatment of IVF-ET [10, 11], which can regulate the hormone level of patients, coordinate the development of endometrium and oosperm, and provide good conditions for the implantation so as to increase patients' pregnancy rate. After implantation of oosperm, progesterone can also inhibit the myometrium from shrinking, reduce the excitability of uterine smooth muscle, and reduce its sensitivity to oxytocin for a better environment for embryo growth.

The article "Clinical Efficacy of Assisted Reproductive Technology Combined with Progesterone Capsules in the Treatment of Infertility Caused by Diminished Ovarian Reserve and Its Influence on Serum FSH, E2, and LH Levels of Patients" was retracted in 2023. Reason: concerns about the peer review.

At present, there is no study on the combination of IVF-ET and progesterone in the treatment of infertility caused by DOR. In order to improve the application efficiency of progesterone, progesterone capsules were selected as the auxiliary drug in this study to explore the practical effect of IVF-ET and progesterone on infertility caused by DOR. The results are as follows.

## 2. Materials and Methods

### 2.1. General Data

The data of 120 patients with infertility caused by DOR admitted to our hospital (February 2019–February 2020) were retrospectively analyzed. Inclusion criteria were as follows: (1) patients and their families fully understood the research process and signed the consent form. (2) After examination, patients met the diagnostic criteria of DOR in *Gynecology* [12]; that was, patients were under the age of 40 and suffered from amenorrhoea for 3 months, with FSH levels above 10 U/L, E_2_ levels below 50 ng/L, and LH levels above 2 U/L. (3) Hysterosalpingogram (HSG) showed that oviducts were unobstructed bilaterally. (4) Antral follicle count (AFC) was 5 or below examined by vaginal B-ultrasonography in the natural period. Exclusion criteria were as follows: (1) patients had mental problems or could not be communicated with. (2) Patients had PCOS, hyperprolactinemia, malignant tumors, and endometrial hyperplasia. (3) Patients suffered from infertility due to oviduct or quality of semen and secondary amenorrhea due to organic lesions of the uterus. (4) Patients had contraindications to hormone treatment. (5) Patients received hormone treatment in recent 3 months. (6) Patients underwent oophorectomy.

A total of 120 patients were equally divided into the experimental group and the control group according to the order of admission. In the experimental group, the age of the patients was between 24 and 39 years old, with an average age of (32.54 ± 2.14) years. The course of infertility was (5.56 ± 1.65) years. The BMI was (23.21 ± 1.22) kg/m^2^. Among them, 22 patients had a monthly income of more than 5000 yuan, and 40 patients had educational degree of high school or above. In the control group, the age of the patients was between 25 and 38 years old, with an average age of (32.56 ± 2.10) years. The course of infertility was (5.41 ± 1.60) years. The BMI was (23.20 ± 1.24) kg/m^2^. Among them, 21 patients had a monthly income of more than 5000 yuan, and 41 patients had educational degree of high school or above. No significant difference was found in the general data of patients between both groups (*P* > 0.05), and the study was approved by the Hospital Ethics Committee.

### 2.2. Withdrawal Criteria

Withdrawal criteria were as follows, and the examination results of patients were not analyzed. (1) Patients experienced adverse events or serious adverse events and were inappropriate to continue the experiment. (2) Patients appeared to deteriorate during the experiment and were inappropriate to continue the experiment according to the doctor's judgement. (3) Patients had severe complications and special physiological changes and were inappropriate to continue the experiment according to the doctor's judgement. (4) Patients were not willing to continue during the experiment and asked the research group for withdrawal.

### 2.3. Methods

All patients underwent IVF-ET and were treated with short-acting diphereline for a long term. Patients were taking 0.1 mg of short-acting dafirin in the midluteal phase and 1 week before treatment (Chengdu Tiantai Mount Pharmaceutical Co., Ltd., NMPA approval No. H20058648) till menstruation (days 3–5) for measurement of FSH, E_2_, and LH levels. Then, patients were examined by a color Doppler ultrasound (GE Healthcare, color ultrasound diagnostic instrument, Voluson P6, NMPA Certified No. 20152062178) and given human chorionic gonadotropin (HCG) (ACON Biotech Hangzhou Co., Ltd., NMPA approval No. S20003013) when pituitary was in a sensitive status, B-ultrasound showed no follicular cysts, and the endometrial thickness was within 5 mm. B-ultrasound was performed 5 days after taking drugs. When the largest follicle reached 20–22 mm, patients were given 7000–10000 IU of HCG, and ultrasound-guided transvaginal oocyte retrieval was performed after 36 h. According to patients' condition, IVF or fertilization of microinjection of a single spermatozoon in follicular plasma was performed, and the embryo was scored in pronuclear and cleavage stage. ET was performed on the second day after oocyte retrieval, and the transferred cells were M-II oocytes with a maximum value of 2.

The article "Clinical Efficacy of Assisted Reproductive Technology Combined with Progesterone Capsules in the Treatment of Infertility Caused by Diminished Ovarian Reserve and Its Influence on Serum FSH, E2, and LH Levels of Patients" was retracted in 2023. Reason: concerns about the peer review.

The experimental group was treated with progesterone capsules at the same time. Patients received progesterone capsules (Zhejiang Xianju Pharmaceutical Co., Ltd., NMPA approval No. H20041902) orally from the 16th day of menstruation for 10 d, 200 mg daily, 21 d as one period, for a total of three periods.

### 2.4. Observation Criteria

1. Ovarian-related indexes: before and after treatment, the blood perfusion of the ovarian artery of patients was observed by a laser Doppler flowmetry (GE Healthcare, color ultrasound diagnostic instrument, Voluson P6, NMPA Certified No. 20152062178), and the blood flow signal was probed at the hilum of the ovary, the follicular wall, and the corpus luteum. Peak systolic velocity (S), end-diastolic velocity (D), peak systolic velocity of the ovarian artery (PSV), and endometrial thickness were recorded. The pulsatility index (PI), resistance index (RI), ovarian average volume (OAV), and S/D were calculated.
2. Follicular development: ovulation of patients was monitored by B-ultrasound, and the ovulation signs were the collapse of the dominant follicle, the disappearance of anechoic areas of follicles with a clear outline, and the presence of effusion in the pelvic cavity. The days of ovulation induction, the number of M-II oocytes, the number of fertilized M-II oocytes, AFC, the thickness of endometrium on the day of ovulation, and the number of high-quality embryos were recorded. The evaluation criteria of high-quality embryos were as follows. The embryo was scored in the pronuclear and cleavage stages. As 7–10 blastomeres in uniform shape were observed the day after oocyte retrieval and fragments were under 5%, it was considered as a first-class embryo. As fragments were between 5% and 20%, it was considered as a second-class embryo. The first-class and second-class embryos were high-quality embryos.
3. Serum hormone levels: before and after treatment and on the second day of menstruation, 5 ml of fasting cubital venous blood was drawn from patients for measurement of serum FSH, E_2_, and LH levels by electrochemiluminescence immunoassay (Cobas e411 electrochemiluminescence instrument with matching reagent, NMPA Certified No. 2011 3402843).
4. Pregnancy outcomes: the clinical pregnancy rate, abortion rate, and multiple births rate were compared.

The article "Clinical Efficacy of Assisted Reproductive Technology Combined with Progesterone Capsules in the Treatment of Infertility Caused by Diminished Ovarian Reserve and Its Influence on Serum FSH, E2, and LH Levels of Patients" was retracted in 2023. Reason: concerns about the peer review.

### 2.5. Statistical Processing

In this study, the data were processed by SPSS20.0 and graphed by GraphPad Prism 7 (GraphPad Software, San Diego, USA). Including enumeration data and measurement data, the study used *X*^2^ test and *t*-test. The differences were statistically significant at *P* < 0.05.

## 3. Results

### 3.1. Comparison of Ovarian-Related Indexes

Compared with the control group, ovarian-related indexes of the experimental group were obviously better after treatment (*P* < 0.001) (see Figure 1).

### 3.2. Comparison of Follicular Development

Compared with the control group, follicular development of the experimental group was obviously better after treatment (*P* < 0.001) (see Table 1).

### 3.3. Comparison of Serum Hormone Levels

In the experimental group, the FSH level was (5.99 ± 1.20) U/L, the E_2_ level was (540.12 ± 3.54) ng/L, and the LH level was (3.10 ± 0.35) U/L after treatment, which was significantly better than those of the control group (*P* < 0.001; Table 2).

### 3.4. Comparison of Pregnancy Outcomes

Compared with the control group, the clinical pregnancy rate of the experimental group was obviously higher (*P* < 0.05), and the abortion rate of the experimental group was obviously lower (*P* < 0.05), with no significant difference in multiple births rate between both groups (*P* > 0.05), see Figure 2.

## 4. Discussion

With increasing age, the function of ovarian interstitial cells decreases, and the microenvironment in the body is gradually unbalanced, which affects follicular development. In addition, hormone disorders of the ovary are triggered by a lot of factors, such as the faster pace of modern life, more stimulation on the hypothalamus, hypophysis, and ovary, and reduced secretion rate of immunocompetent substances. Therefore, the incidence of DOR is increased [13–15]. Clinical studies show that patients with DOR often present with abnormal serum FSH, E_2_, and LH levels and decreased AFC. Severe cases even have amenorrhea and ovarian function decline, leading to a higher incidence of infertility caused by DOR [16, 17]. At present, women's delayed childbearing has become a trend of population development. More patients with infertility caused by DOR resort to IVF-ET treatment [18], but DOR patients are prone to have poor ovarian response during IVF-ET treatment; that is, patients have low sensitivity to Gn in the process of controlled ovulation induction, resulting in increased Gn dose. However, the number of ovum obtained in each treatment period of patients has not been significantly improved, and the oocytes are still low quality. After fertilization, embryos are of poor quality and hard to implant, and some pregnant patients still have a high abortion rate and a low probability of successful delivery [19]. Once the pregnancy fails, patients will receive further treatment. The long treatment time and the high cost exert mental pressure on patients, which is not conducive to their further treatment. Therefore, it is the focus of IVF-ET treatment for infertility caused by DOR to find effective ways to improve embryo quality and implantation rate.

The article "Clinical Efficacy of Assisted Reproductive Technology Combined with Progesterone Capsules in the Treatment of Infertility Caused by Diminished Ovarian Reserve and Its Influence on Serum FSH, E2, and LH Levels of Patients" was retracted in 2023. Reason: concerns about the peer review.

Progesterone has been used for 10 years in IVF-ET treatment in China [2]. The reason is that GnRH-a used in IVF-ET treatment causes poor hypothalamic-pituitary function and affects progesterone secretion in the luteal phase, and an abnormal ratio of estrogen and progesterone will lead to progesterone deficiency. Meanwhile, progesterone auxiliary treatment can improve the secretory reaction of the endometrium, accelerate the growth rate of the endometrial gland in the latter period of menstruation, and increase uterine blood supply and thicken endometrium, making preparations for implantation of fertilized ovum [20]. Therefore, this study showed that, compared with the control group, the thickness of endometrium after treatment and on the day of ovulation and the ovarian hemodynamic indexes of the experimental group were conspicuously improved, which confirmed that progesterone had a high supportive function and could provide good conditions for embryo implantation. Previous studies have shown that progesterone injection into rats with infertility caused by DOR can regulate their FSH, E_2_, and LH levels [21]. This study also obtained the same results that after IVF-ET and progesterone treatment, serum hormone levels of both groups were improved, indicating the improvement of patients' follicular growth and development and recovery of ovulation capacity. Therefore, the ovarian-related indexes and follicular development were better than those before treatment, and the data of the experimental group were better than those of the control group.

The article "Clinical Efficacy of Assisted Reproductive Technology Combined with Progesterone Capsules in the Treatment of Infertility Caused by Diminished Ovarian Reserve and Its Influence on Serum FSH, E2, and LH Levels of Patients" was retracted in 2023. Reason: concerns about the peer review.

Moreover, progesterone treatment further increased the rate of endometrial gland proliferation from proliferative to secretory phase, so the clinical pregnancy rate in the experimental group was significantly higher than that in the control group (*P* < 0.05). After the implantation of fertilized ovum, progesterone could reduce the excitability of uterine smooth muscle, inhibit uterine contraction and immune reaction, and prevent maternal rejection for the fetus [22, 23], thus ensuring the early growth of the fetus. Therefore, compared with the control group, the abortion rate in the experimental group was obviously lower (*P* < 0.05). It is worth noting that no obvious difference was found in the multiple births rate between both groups (*P* > 0.05), indicating that single birth and multiple births could not be affected by progesterone. In the study of Kim et al. which applied IVF-ET and progesterone in patients with infertility caused by PCOS and endometriosis, it also found that this treatment method could not affect the multiple births rate but affected the clinical pregnancy rate [24].

In conclusion, ART combined with progesterone capsules can improve the serum hormone levels, ovarian function, follicular development, and clinical pregnancy rate for patients with infertility caused by DOR, which should be applied in practice.

## Figures and Tables

**Figure 1:** Comparison of ovarian-related indexes $\left(\bar{x}\pm s\right)$ (^*∗*^Note: in Figure 1, the abscissa was before and after treatment from left to right, respectively. The black area indicated the experimental group, and the gray area indicated the control group. ^#^ indicated *P* < 0.001). (a) PI. No significant difference was found in PI between both groups before treatment (1.49 ± 0.21 vs 1.50 ± 0.23, *P* > 0.05). After treatment, compared with the control group, PI of the experimental group was obviously higher (2.34 ± 0.35 vs 1.87 ± 0.25, *P* < 0.001). (b) RI. No significant difference was found in RI between both groups before treatment (0.90 ± 0.11 vs 0.91 ± 0.12, *P* > 0.05). After treatment, compared with the control group, RI of the experimental group was obviously lower (0.68 ± 0.10 vs 0.78 ± 0.12, *P* < 0.001). (c) OAV. No significant difference was found in OAV between both groups before treatment (3.98 ± 0.35 vs 3.96 ± 0.36, *P* > 0.05). After treatment, compared with the control group, OAV of the experimental group was obviously higher (6.05 ± 0.45 vs 5.10 ± 0.45, *P* < 0.001). (d) S/D. No significant difference was found in S/D between both groups before treatment (3.00 ± 0.24 vs 3.02 ± 0.28, *P* > 0.05). After treatment, compared with the control group, S/D of the experimental group was obviously lower (2.10 ± 0.12 vs 2.58 ± 0.20, *P* < 0.001). (e) PSV. No significant difference was found in PSV between both groups before treatment (0.79 ± 0.15 vs 0.78 ± 0.14, *P* > 0.05). After treatment, compared with the control group, PSV of the experimental group was obviously higher (2.29 ± 0.20 vs 1.85 ± 0.23, *P* < 0.001). (f) Thickness of endometrium. No significant difference was found in the thickness of the endometrium between both groups before treatment (3.55 ± 0.14 vs 3.59 ± 0.15, *P* > 0.05). After treatment, compared with the control group, the thickness of the endometrium of the experimental group was obviously higher (5.01 ± 0.26 vs 4.66 ± 0.19, *P* < 0.001).

The article "Clinical Efficacy of Assisted Reproductive Technology Combined with Progesterone Capsules in the Treatment of Infertility Caused by Diminished Ovarian Reserve and Its Influence on Serum FSH, E2, and LH Levels of Patients" was retracted in 2023. Reason: concerns about the peer review.

**Figure 2:** Comparison of pregnancy outcomes (*n* (%)). (^*∗*^Note: in Figures (a, b, c), the experimental group was on the left, and the control group was on the right. ^#^ indicated *P* < 0.001. (a) Clinical pregnancy rate. The black area was pregnancy, and the gray area was not pregnancy. Compared with the control group, clinical pregnancy rate of the experimental group was obviously higher (35 vs 24, *P* < 0.05). (b) Abortion rate. The black area was abortion, and the gray area was not abortion. Compared with the control group, abortion rate of the experimental group was obviously lower (4 vs 8, *P* < 0.05). (c) Multiple births rate. The black area was multiple births, and the gray area was single birth, with no significant difference in multiple births rate (6 vs 4, *P* > 0.05)).

**Table 1:** Comparison of follicular development $\left(\bar{x}\pm s\right)$.

Group	Experimental group (*n* = 60)	Control group (*n* = 60)	*X* ^2^/*t*	*P*
Days of ovulation induction (d)	18.21 ± 3.21	12.54 ± 3.41	9.378	<0.001
Number of M-II oocytes				
Total	210	180		
Average	5.10 ± 1.11	3.54 ± 1.23	7.293	<0.001
Number of fertilized M-II oocytes	3.98 ± 0.65	3.00 ± 0.54	8.983	<0.001
Antraol follicle count	4.35 ± 0.41	3.10 ± 0.35	17.961	<0.001
Thickness of endometrium on the day of ovulation (mm)	10.10 ± 1.26	8.00 ± 1.35	8.809	<0.001
Number of high-quality embryos	1.85 ± 0.35	1.10 ± 0.23	13.871	<0.001
Gn dosage (U)	1765.68 ± 554.21	2298.65 ± 558.65	5.246	<0.001

**Table 2:** Comparison of serum hormone levels $\left(\bar{x}\pm s\right)$.

Indexes	Experimental group		Control group		*t*	*P*
FSH	Before treatment	20.10 ± 3.54	Before treatment	20.54 ± 3.21	0.713	0.477
(U/L)	After treatment	5.99 ± 1.20	After treatment	10.22 ± 2.54	11.664	<0.001
	*t*	29.240	*t*	19.529		
	*P*	<0.001	*P*	<0.001		

E_2_	Before treatment	100.65 ± 6.98	Before treatment	101.68 ± 6.12	0.859	0.392
(ng/L)	After treatment	40.12 ± 3.54	After treatment	49.68 ± 3.68	14.502	<0.001
	*t*	59.908	*t*	46.404		
	*P*	<0.001	*P*	<0.001		

LH	Before treatment	16.45 ± 2.54	Before treatment	16.87 ± 2.58	0.899	0.371
(U/L)	After treatment	3.10 ± 0.35	After treatment	7.98 ± 1.23	29.559	<0.001
	*t*	40.331	*t*	24.093		
	*P*	<0.001	*P*	<0.001		

The article "Clinical Efficacy of Assisted Reproductive Technology Combined with Progesterone Capsules in the Treatment of Infertility Caused by Diminished Ovarian Reserve and Its Influence on Serum FSH, E2, and LH Levels of Patients" was retracted in 2023. Reason: concerns about the peer review.

## Data Availability

The data used to support the findings of this study are available on reasonable request from the corresponding author.
